# Genetic algorithm optimization of heliostat field layout for the design of a central receiver solar thermal power plant

**DOI:** 10.1016/j.heliyon.2023.e21488

**Published:** 2023-11-01

**Authors:** Muhammad Haris, Atiq Ur Rehman, Sheeraz Iqbal, Syed Owais Athar, Hossam Kotb, Kareem M. AboRas, Abdulaziz Alkuhayli, Yazeed Yasin Ghadi, Kitmo

**Affiliations:** a Department of Electrical Engineering, Balochistan University of Information Technology, Engineering and Management Sciences (BUITEMS), Quetta 87300, Pakistan; b Department of Electrical Engineering, University of Azad Jammu and Kashmir, Muzaffarabad, Pakistan; c Department of Electronic Engineering, Balochistan University of Information Technology, Engineering and Management Sciences (BUITEMS), Quetta 87300, Pakistan; d Department of Electrical Power and Machines, Faculty of Engineering, Alexandria University, Alexandria 21544, Egypt; e Electrical Engineering Department, College of Engineering, King Saud University, Riyadh 11421, Saudi Arabia; f Department of Computer Science and Software Engineering, Al Ain University, Abu Dhabi 15322, United Arab Emirates; g University of Maroua, National Advanced School of Engineering of Maroua, Department of Renewable Energy, P.O. Box 46 Maroua, Cameroon

**Keywords:** Security distance, tower height, Length ratio, Length of heliostats

## Abstract

The heliostat field layout in a central receiver solar thermal power plant has significant optical losses that can ultimately affect the overall output power of the plant. In this paper, an optimized heliostat field layout based on annual efficiency and power of 50 MW for the local coordinates of Quetta, Pakistan, is proposed. The performance of two different heliostat field layouts such as radial staggered and Fermat's spiral distribution are evaluated and different design points in a year are considered for the analysis. The field layouts are then optimized using a rejection sampling based Genetic Algorithm (GA). It considers the output power and mean overall efficiency for vernal equinox, summer solstice, autumnal equinox, and winter solstice as objective functions. The GA optimizes the heliostat field parameters, namely, security distance (DS), tower height (TH), heliostat width to length ratio (WR), and the length of heliostats (LH). The study system was developed in MATLAB for validation. It was observed that for the radial staggered layout, the number of heliostats decreased by 364 and the efficiency was improved by 8.52 % using GA optimization relative to unoptimized results field layout. The annual efficiency for Fermat's spiral configuration was improved by 14.62 % and correspondingly, the number of heliostats decreased by 434.

## 1 Introduction

### 1.1 Background and motivation

Concentrated solar thermal power (CSP) is an emerging technology to generate clean electrical energy. The idea of such systems was first proposed in 1957 [1]. These plants can be used in combination with other technologies to provide flexibility and better economic benefits to the national grid [2]. Salient features like thermal energy storage (TES) and equipment sharing are among the vital characteristics of CSP that add to their importance. These plants are also proven to be very cost-effective among their other counterparts to generate clean electrical energy at a large scale, which further advocates their inclusion in a country's power generation block [3].

The heliostat field layout greatly influences the overall functioning of CSP. The width, height, and length of the heliostat, cosine efficiency, and other factors like shading and blocking of heliostat mirrors, and flux spillage account for about 50 % of the total losses and 40 % of the total costs in the plant [4]. The arrangement of heliostats around a tower is also associated with the operational losses of the plant. This necessitates the design of an optimized heliostat field to reduce these losses and correspondingly the land usage. Efficient heliostat fields also minimize the environmental impact associated with the power generation [5]. Accordingly, numerous studies have been proposed in the literature which consider these attributes to increase the overall output that can be extracted from a particular heliostat field.

### 1.2 Literature review

The power generation in central receiver power plant is greatly affected by the performance of heliostat field. The field performance evaluation is based on various parameters which include evaluation of overall efficiency, heliostat tracking and focusing etc. This section provides the detailed work related to the design and optimization of heliostat field layout.

The overall field efficiency is typically a function based on cosine losses, shading and blocking, atmospheric attenuation, and spillage factor. For the evaluation of overall efficiency of heliostat field, an “Error Cone” simulation model was presented by Ref. [6]. In Ref. [7], the annual energy calculation was made for a predefined heliostat field. Similarly, based on the output power and yearly normalised energy surfaces, a method for the generation of heliostat fields was proposed in Ref. [7]. The analytical modelling for heliostat field layout considering the blocking factor of 1 was presented in Ref. [8]. The optimization of field efficiency of power plant in Dagget was presented in Ref. [9]. Similar study based on comparative analysis of different molten salts was presented by the authors in Ref. [8].

A comparison between spiral and radial staggered layouts for PS10 and Gemasolar power plants was made in Ref. [10]. The Spiral is considered better than radial staggered layout because of having better cosine efficiency. Reference [11] designed a heliostat field layout that was based on the format spiral distribution. Their optimization algorithm involved a genetic algorithm in which the heliostats are first distributed and then optimized based on their land usage and distance from the tower. A differential evolution algorithm was proposed for Dhahran, Saudi Arabia in Ref. [12]. The study considered weighted and unweighted insolation normal efficiency. A pattern-free greedy based approach was presented in Ref. [13]. A MATLAB graphical user interface-based program was proposed by Ref. [14] to generate optimized field layouts based on radial cornfield and radial staggered configurations the study considered atmospheric attenuation and cosine efficiency of the field to be optimized.

Levelized cost of electricity (LCOE) was the objective function subject to the tower and field layout constraints which were optimized by the algorithm proposed by Ref. [15]. The levelized cost of electricity is associated with the operational and maintenance losses within a plant. These losses can be mitigated with the help of efficient scheduling techniques as proposed by Ref. [16] which aimed to reduce the site slope effect along with heliostat cleaning which the authors refer to as “de-soiling”. Different algorithms for the optimization of field layout based on the levelized cost of electricity constraint are presented in literature [[17], [18], [19]].

Ray tracing methods for optimization of heliostat field generating 400–550 kW power were presented in Ref. [20]. In the study, solar radiation was first estimated and then analyzed for two differently sized heliostats. An oversized field can be made efficient with the help of polygon optimization and boundaries [[18], [19], [20], [21]]. Blocking and shadowing are two of the most important factors determining the field efficiency; they are also computationally expensive [21]. Analytical geometry methods are presented in the literature to find the problem heliostats, and results are compared with other methods to reduce the computational time [22,23].

The calibration and installation of heliostats is another optimization variable which has been considered by different studies in their objective functions. Heliostats within a field must be capable of tracking the sun throughout the year. The post installation calibration is therefore necessary as presented and optimized by Ref. [24]. Deep-learning and different image processing-based algorithms have also been implemented for control and tracking of heliostats [25,26]. Central receiver systems, therefore, can be modeled as power generating structures having multiple modules efficiency of each of which is directly or indirectly linked with the overall output power of the plant. Hence, the total generated output power is taken as a fitness constraint in this study.

### 1.3 Paper organization

The structure of this study is designed in the following manner. In Section 1, a summary of the important field layout constraints that were considered during optimization by different studies and their respective optimization strategies is presented. Section 2 illustrates the methodology of designing the optimized heliostat field layout for central receiver power plant development in Quetta, Balochistan. Section 3 describes the performance analysis of field layout before and after optimization. The results and conclusion are presented in Section 4. Finally, the paper is concluded in Section 5.

## 2 Methodology

### 2.1 Brief description of work

In this study, a heliostat field layout is designed for developing Central Receiver Solar Thermal Power Plant with capacity of 50 MW in Quetta, Balochistan. The designed system is then optimized using Genetic Algorithm. The study system is developed in MATLAB for analysis. The two different techniques used for the design of heliostat field layout are Radial Staggered and Fermat Spiral Distribution. In addition, the performance of the two heliostat field layout techniques (i.e., Radial Staggered and Fermat Spiral Distribution) considering the output power, magnitude and optical efficiency is investigated. In the following section, the design of heliostat field layout and genetic algorithm are illustrated in detail. It must be noted that alternative optimization tools like SolarPILOT, System Advisor Model (SAM) and other programs provide a very detailed economic model for optimization and design of such power plants. However, this study is based on leveraging the data specifically acquired from the design point location coordinates. It can be considered as the very first feasibility study for assessment of concentrating solar thermal potential in Quetta, Balochistan. Therefore, the algorithm developed here does not claims to be competing with existing tools and all the results presented here are in relation with the unoptimized layouts. However, more advanced version of these algorithms is being developed for further enhancement of these works.

### 2.2 Description of the design point location

The system is designed to analyse the feasibility and solar thermal power potential of Quetta, Balochistan which is in Pakistan with the GPS coordinates of 30.1798° N, 66.9750° E. The locality has a rich solar potential with an average DNI ranging in between 1500 and 2750 W/m^2^/day throughout the year [27]. In 2015, a meteorological station was installed for the real time DNI measurement of solar insolation [28]. The site location along with overview are shown in Fig. 1, Fig. 2, respectively. The Tier 2 meteorological data acquisition system shown in Fig. 3 logged data at 10 min intervals. The same data has been utilized in the design and analysis of 50 MW central receiver solar thermal power generation system in Quetta, Balochistan.

**Fig. 1:** Location of Fatima Jinnah Girls hostel, BUITEMS.

**Fig. 2:** Site overview of the hostel building rooftop at BUITEMS, Quetta [28].

**Fig. 3:** Data acquisition system installed at the rooftop of a hostel in BUITEMS, Quetta [28].

### 2.3 Design of heliostat field layout

In the designing of field layouts, various constraints are considered. The shading, blocking, intercept, cosine effect, atmospheric attenuation, plant maintenance and outages mentioned in Refs. [28,29] receiver thermal efficiency as mentioned in Ref. [30] and other factors presented accordingly are considered. Therefore, in this study, field layouts for different design parameters are proposed and optimized. In the first part, heliostat field layouts based on both radial staggered, and Fermat's spiral arrangement are designed and compared based on their optical and annual performance. Steps involved in the implementation of this procedure are explained in the succeeding articles.

### 2.4 Heliostat field layout modelling based on radial staggered configuration

In this heliostat field layout, the radially staggered heliostats are arranged in the form of concentric circles (Fig. 4) [31]. The centre of the field contains the receiver or tower on which the solar energy is concentrated. The radial distance is calculated from the same position. As the radial distance from the tower increases, distance between adjacent heliostats is also increased. This helps the heliostats get maximum freedom while rotating horizontally and vertically. The position of each heliostat can be mapped as an x and y coordinate on a cartesian coordinate plane as shown in Fig. 4. The first ring comprising of heliostats in any heliostat field is called “essential ring” [32]. This ring is followed by the ring called “staggered ring”. Heliostats in this type of field layout are placed in a particular ring and the radial distance is increased until another heliostat can be placed in between two adjacent heliostats. Once this constraint is reached, the radial distance value is reset to a new azimuthal angle and a new.

**Fig. 4:** Radial staggered field layout.

group of heliostats is started. The equations which govern the radial distance and azimuthal angle along with other important variables are explained as follows.

The x and y coordinates of the field layout are calculated by using the transformation of cartesian coordinates into circular cylindrical coordinate systems as shown in Equation (1) [33].

(1) $$e_{1}=R_{Zone}\;\mathrm{Cos}\;\varphi n_{1}=R_{Zone}\;\mathrm{Sin}\;\varphi z_{1}=z$$

Where, $R_{zone}$ = radius of the ring and *φ* = Azimuthal Spacing between adjacent heliostats. The radial spacing between two rings is analytically expressed in Equation (2) [33]:

(2) $$\Delta R=HM\left(1.44\;\cot\left(\theta_{L}\right)-1.094+3.068\theta_{L}-1.1256{\theta_{L}}^{2}\right)$$

Equation (3) gives the azimuthal spacing between two mirrors.

(3) $$\Delta A=WM\left(1.749+0.6396\theta_{L}\right)+\frac{0.2873}{\theta_{L}-0.04902}\;\left(m\right)$$

Where *θ*_*L*_ is the altitude angle, which is different for each heliostat. It is a function of the radial distance between the central tower and the heliostat point of interest, its value is determined using Equation (4):

(4) $$\theta_{L}=\tan^{-1}\left(\frac{1}{r}\right)\;\left(\deg\right)$$

Where r is the radial distance of the heliostat from the tower and is measured as a function of tower heights. This radius is very crucial for determining cosine efficiency whose value can be determined using Equation (5) as defined in Ref. [33].

(5) $$\cos\;2\theta_{i}=\frac{\left(z_{o}-z_{1}\right)\sin\left(\alpha \right)-e_{1}\;\cos\left(\alpha \right)\sin\left(A\right)-n_{1}\;\cos\left(\alpha \right)\cos\left(A\right)}{{\left[{\left(z_{o}-z_{1}\right)}^{2}+{e_{1}}^{2}+{n_{1}}^{2}\right]}^{1/2}}$$

Where alpha and A are the angles of elevation and azimuth of the sun. These two angles change their direction throughout the day depending upon the sun's location and hour. In terms of latitude φ and solar hour angles ω, these functions are represented using Equation (6).

(6) $$\alpha =\sin^{-1}\left(\sin\;\delta \;\sin\;\varphi +\cos\;\delta \;\cos\;\omega \;\cos\;\varphi \right)$$

Notice that for the calculation of cosine efficiency, the radial staggered and Fermat's spiral distribution follow the same Equation. In Ref. [31], a mathematical model was presented that included an algorithm and a c code for generating a radial staggered field layout. The complete step-by-step procedure, as explained below, can be applied easily on a field having radially staggered heliostats to achieve a blocking factor equal to 1. Steps for implementation involve.

- Location of field dimensions on a cartesian coordinate plane: The heliostat in this method of generation is represented as a circle (Fig. 4).
- The diameter of this circle as seen from above, is equal to the heliostat diagonal. This is done to reduce the heliostat collisions while tracking the sun along the azimuth or the altitude.
- The radius of the first row of heliostats should equal tower heights.

The algorithm presented in the methodology section was practically checked and implemented using MATLAB for the design point location and latitude.

### 2.5 Heliostat field based on Fermat's spiral distribution

Another method for generating a heliostat field is the Fermat spiral configuration [34,35]. It is based on the natural growth of sunflower heads, also known as "capitula" (Fig. 5, Fig. 6). This distribution follows a pattern of two sets of arcs. One running in each direction from clockwise to counterclockwise.

**Fig. 5:** Shape of a typical sunflower head.

**Fig. 6:** Fermat's spiral distribution.

The patterns follow Equation (7) based on circular coordinate system.

(7) $$r=c\sqrt{n}\theta =137.508n$$

Where r is the position vector magnitude, c is a scaling factor, and n is the index number. θ is the azimuthal angle of the coordinates.

Considering the location of heliostats as x and y coordinates on a cartesian plane these equations can be easily transformed into the corresponding coordinate system as shown in Equation (8).

(8) x=rcos(θ)y=rsin(θ)

After both the field layouts are generated for predefined parameters, optimization is started by taking this initial layout as a "Seed Heliostat Field." This task is performed using the Genetic Algorithm as defined.

## 3 Optimization of field layout

The genetic algorithm is an evolutionary algorithm used for optimizing problems with non-linear or complex solutions. It is basically applied where many factors influence the performance of a single objective function. Inspired by Charles Darwin's theory of evolution, the algorithm finds ways to reproduce individuals that are the fittest in a generation. Instead of starting from a single guess, the algorithm starts with a population of guesses, which is random in nature and evolves over generations or iterations. One of the most unique features of a GA is that all the unimportant and obsolete solutions from the solution set are eradicated in the mutation and crossover step. Various research works have focused on the improvement of this step since any GA convergence is based on it. A non-uniform or awful crossover can lead to a non-local and non-optimal solution that is not desired in such algorithms. Fig. 7 shows the steps involved in implementing the genetic algorithm. If the termination criteria are not met, the algorithm starts another iteration which calculates the fitness of evolved chromosomes and tries to make the solution more compact and optimized. All the steps used in the GA which were performed in this work to optimize the heliostat field layout are explained in the following sections.

**Fig. 7:** Flowchart for the implementation of genetic algorithm.

### 3.1 Population initialization

The initial population in a genetic algorithm consists of a random set of solutions that are independent of each other. Each set is called a "Chromosome," and the parameter to be optimized is known as a "Gene." The objective of implementing a genetic algorithm is to find the fittest genes possible to solve the problem at hand. Therefore, mathematically, it can be expressed using Equation (9) as follows:

(9) Chromosome=[p1,p2,p3,p4]

### 3.2 Tower height (TH)

This is the height of the receiver tower taken in meters. The field efficiency and overall economics of the plant are dictated to a great extent by this parameter. Tower height is a function of the weight of the receiver. Steel structures are preferred for tower heights less than 120 m; however, concrete structures are made for larger towers. According to the research conducted by Sterns Rogers engineering company [34], tower heights between 50 and 300 m are economical. Therefore, the same range is taken as a constraint for optimization in this study.

### 3.3 Length of heliostat (LH)

The effective area of heliostat determines the magnitude of solar flux which is incident on them. Correspondingly, it determines the input power and incident efficiency of plant. According to Ref. [30], this area lies between 25 and 150 m^2^. Therefore, this constraint has been set in the range of 5–20 m.

### 3.4 Security distance between heliostats (DS)

Modern solar fields incorporate heliostats that track the sun throughout the day using steppers and servo motors specially designed electrical to mechanical energy transducers [35]. They have an input and output feedback mechanism for checking the current heliostat angle. The heliostats move around their axis in a circular pattern which makes them prone to collision with other heliostats near them. To cater for this, a security distance should be present between heliostats in the same row and group. A factor called "security distance" is used to mathematically compensate this error-inducing situation. This distance is kept in the range of 0.1–0.5 [36].

### 3.5 Heliostat width to length ratio (WR)

This ratio affects the cosine efficiency and field placement efficiency of the heliostat. Its range is kept between 1 and 2. The previously explained four articles complete our genes of a chromosome used in population initialization. The chromosomes are depicted in tabulated form in Table 1. Based on these ranges, the population of 30 individuals is first initialized, and their fitness is calculated. After that, the tournament selection method is used for the selection of parents to complete the crossover step.

**Table 1:** Chromosome in this problem.

Chromosome with Defined Ranges of Genes			
Tower Height *(TH)*	Length of Heliostat *(LH)*	Heliostat Width to Length Ratio *(WR)*	Security Distance between heliostats *(DS)*
50–300 m	5–20 m	1–2	0.1–0.5 m

### 3.6 Fitness function

The fitness function in our problem is the power generated by each heliostat and its overall efficiency. The total efficiency of the field is the average efficiency of all heliostats. Thus, mathematically, the fitness function is divided into two parts. The first part is power generated by an individual heliostat. It is given by Equation (10) as follows:

(10) $$Power\;Generated\;by\;Each\;Heliostat=I\rho \cos\;\omega \;f_{sp}f_{sb}\;f_{at}\;\left(\frac{W}{m^{2}}\right)$$

Where I = Design Point DNI and ρ(themirrorreflectivityco−efficient)=0.88 based on [37].

Similarly, the second part of the fitness function in our problem is given in Equation (11) as follows:

(11) $$Overall\;Efficiency\;of\;Field=\cos\;\omega \;f_{b}\;f_{sp}f_{at}$$

Where $f_{b}$ is the blocking factor and is taken as 0.97 in this problem due to its reduced effect on the overall field efficiency. fsp is the spillage factor [38] and is given using Equation (12):

(12) $$f_{sp}=\frac{PH\left(wr.\frac{LH}{2\sqrt{2}\sigma_{r}},-a_{r},a_{r}\right)\times PH\left(\frac{LH}{2\sqrt{2}\sigma_{r}},-a_{r},a_{r}\right)}{a_{r}^{2}}$$

Where $a_{r}=\frac{\sqrt{A_{h}}}{2\surd 2\sigma_{r}}$ and σr = Dispersion of effective sun-shape. To cater for its random nature, a gaussian approximation for this parameter is considered by taking its value as 2.51 mrad in this study. The value for PH as a function is given in Equation (13) as follows:

(13) $$PH\left(\xi_{r},-a_{r},a_{r}\right)=\frac{1}{2}\left\{\left(\xi_{r}+a_{r}\right)\mathrm{erf}\left(\xi_{r}+a_{r}\right)+\frac{1}{\sqrt{\pi }}\exp\left[-{\left(\xi_{r}+a_{r}\right)}^{2}\right]-\left(\xi_{r}-a_{r}\right)\mathrm{erf}\left(\xi_{r}-a_{r}\right)-\frac{1}{\sqrt{\pi }}\exp\left[-{\left(\xi_{r}-a_{r}\right)}^{2}\right]\right\}$$

The value of fat is given using Equation (14) as follows [41]:

(14) $$\tau_{a}=0.99326-0.1046S+0.017S^{2}-0.002845S^{3}$$

### 3.7 Keeping and discarding individuals based on their fitness

After the population's generation, each chromosome's fitness is determined, and the sets are sorted out based on the highest efficiency. The first 15 sets with the highest fitness are saved, and the other 15 members of the population are discarded, making way for the offspring of the fittest parents. Mating pool creation based on rejection sampling is used in this study. Rejection sampling is a method of filling up the mating pool based on fitness value of an individual in the population from which it is being selected. The higher the fitness value, higher remains its likeliness to be selected. In short, if an individual has a fitness value of 100 and the maximum fitness is also 100, then, this chromosome has a 100 % chance of being picked up as a parent for mating.

### 3.8 Crossover

The crossover step is initiated by the exchange of parameters among selected parents. The number of exchanged and substituted members can be defined using a random number. We call this random number a crossover point (λ), and according to the procedure defined before, its value lies in the following range as represented by Equation (15):

(15) LowerGenePosition≤λ≤UpperGenePosition

Based on the above equation, the lower and upper gene positions in our problem are 0 and 3, respectively. If λ = 1 parents and crossed-over chromosomes are given respectively as in Equation (16):

(16) $$parent1=\left(p_{m1},p_{m2},p_{m3},p_{m4}\right)parent2=\left(p_{d1},p_{d2},p_{m3},p_{m4}\right)crossedover1=\left(p_{m1},p_{d2},p_{m3},p_{m4}\right)crossedover2=\left(p_{m1},p_{m2},p_{m3},p_{m4}\right)$$

In this step, the values of crossing parents are just exchanged, and there isn't any change in the gene value which doesn't induce diversity in the solution. Therefore, a new optimization parameter is calculated using Equation (17):

(17) $$p_{new1}=p_{m\lambda }+\beta \left[p_{m\lambda }-p_{d\lambda }\right]\;p_{new2}=p_{d\lambda }+\beta \left[p_{m\lambda }-p_{d\lambda }\right]$$

Where β is also a random number whose value lies between zero and one. Based on this, the offspring that are calculated are given in Equation (18):

(18) $$offspring1=\left(p_{m1},p_{new1},p_{m3},p_{m4}\right)offspring2=\left(p_{m1},p_{new2},p_{m3},p_{m4}\right)$$

### 3.9 Mutation

This step introduces diversity in the solution space. The step involves changing the values of selected parameters of selected offspring values of selected offspring in the crossover step to reduce the probability of the algorithm to cycle around different localized solutions to problem. A new variable, γ, is introduced in the step with the range between one and four. The variable dictates the calculation of new parameters based on Equation (19):

(19) $$p_{new}=\left(upperlimit_{\gamma }-lowerlimit_{\gamma }\right)*random+lowerlimit_{\gamma }$$

### 3.10 Convergence

Once these steps are performed, the steps are regressed until convergence is found. The condition for convergence in our case is given in Equation (20) as follows:

(20) $$Convergence\;is\;achieved\;if\;and\;only\;if\;\left(eff^{n}-eff^{n-1}<10^{-4}\right)$$

After the convergence is obtained, the algorithm is stopped, and the locally minimized solution is obtained.

## 4 Results and discussion

### 4.1 Radial staggered field layout for the local coordinates of Quetta, Balochistan

Table 2 represents all the constant values used for initial layout generation based on a radial staggered pattern (Fig. 8). The circle around each coordinate has a diameter equal to heliostat width and a security distance is added in the optimization step to avoid collision during the rotation of heliostats. The initial field layout consisted of a total of 864 heliostats which were optimized and decreased in number after using a genetic algorithm. For this layout, atmospheric attenuation and cosine efficiency are analyzed. The atmospheric attenuation is the resistance or hindrance offered to the reflected sun ray as it travels from the reflecting heliostat towards the receiver where the molten salts are present to be heated. It mainly increases with an increase in the distance from the tower as shown in Fig. 9. It is a very important feature dictating the overall efficiency of a heliostat field as it has a direct physical impact on the path taken by the reflected ray as it travels from the surface of heliostat. Since the fraction of mirror area in front of another one is the first and nearest object hindering the path of a reflected ray, a no blocking field layout was required. In Fig. 8, the results obtained by the implementation of [31] using MATLAB are depicted. Notice that the mirrors closest to central receiver have highest efficiency which corresponds to a higher value of individual power generation by a heliostat. This efficiency is independent of the DNI value of a coordinate and is the same for any location. The parameter which is highly dependent on the path taken by the sun and is different for different design points is cosine efficiency which takes different values for different days and time of the year.

**Table 2:** Constant Parameters of Seed Heliostat Field to be designed for Quetta, Balochistan.

Parameter	Value
Design Point Location for DNI Measurement	BUITEMS, Quetta
Equipment for DNI Measurement	Tier 2 Station with Rotating Shadowband Irradiometer
Design point latitude coordinate (Quetta, Pakistan)	30.271
Blocking Factor	0.95
Heliostat Length	10.95 m
Minimum Radius of Field	65 m
Sunshape's Standard Deviation	2.51 mrad
Heliostat Width to Length Ratio	1
Emissivity of Receiver	0.88
Tower Height (THT)	130 m
Heliostat Length	10.95
Input Power	50 MW

**Table 3:** DNI Values for Important days of Solar Year based on DNI values of Quetta, Balochistan [39].

Solar Event	Date	Day No.	Time	DNI Value		Average DNI (W/m^2^) for the Design Point (BUITEMS, Quetta)
				Date	DNI	
Vernal Equinox	March 21	80	11 a.m.	21-03-2015	858.7907	858.47
				21-03-2016	860.7587	
				21-03-2017	855.8775	
Summer Solstice	June 21	172	11 a.m.	21-06-2015	938.9873	965.64
				21-06-2016	958.3664	
				21-06-2017	999.5806	
Autumnal Equinox	September 23	266	11 a.m.	21-09-2015	748.9886	875.71
				21-09-2016	933.7005	
				21-09-2017	944.4501	
Winter Solstice	December 21	355	11 a.m.	21-09-2015	692.5492	856.63
				21-09-2016	948.4788	
				21-09-2017	928.8578	

These values vary throughout the day and year. Therefore, average values on the following days of interest were considered for the calculation of cosine efficiency.

**Fig. 8:** Unoptimized field layout.

**Fig. 9:** Attenuation Efficiency of the layout.

### 4.2 Cosine efficiency of unoptimized layout for the DNI values of Quetta, Balochistan

In solar power calculations, the cosine efficiency of a location of interest is calculated on four crucial days of the year. Solar DNI data for designing the layout was taken from Ref. [40]. This dataset provides solar radiation level information on 10-min average value for Quetta, Pakistan. The measurements were available from 17 to 09–2015 to 1-05-2017.

For simplicity, it was assumed that all heliostats are reflecting all the incident sunlight onto the receiver. Fig. 10 shows the cosine and overall efficiency plots that were obtained on these days. Notice that different days of the year require different numbers of heliostats based on the position of the sun and location of heliostat. For simplicity, it was assumed that the heliostats were arranged in such a way that all the sunlight is being reflected towards the receiver. Hence, the optical error was not explicitly considered in the study. However, even though the study employed a non-blocking field arrangement, a blocking factor of 0.97 was still considered to cater for optical errors of heliostat. Table 4 shows the number of heliostats required on each important day of the year for generation of the same magnitude of power.

**Fig. 10:** Cosine efficiency for unoptimized radial staggered field layout based on 4 different times (design points) of the year (a) vernal equinox, (b) autumnal equinox, (c) winter solstice and (d) summer solstice.

**Table 4:** Number of Heliostats required to produce same magnitude of input thermal power on different days of the year.

Day of the year	Required Number of Heliostats	Mean (Overall Efficiency) (%)	Overall Mean
Vernal Equinox	864	76.5	74.72
Summer Solstice	935	61.0	
Autumnal Equinox	864	76.5	
Winter Solstice	793	84.9	

### 4.3 Heliostat field layout based on Fermat's spiral distribution for the coordinates of Quetta, Balochistan

For the generation of field layout based on Fermat's spiral distribution, initially, a large layout, approximately five times the actual layout required for generating a given power magnitude, is generated. This large size of the layout is reduced during the optimization step. The attenuation efficiency of this layout is given in Fig. 11. Since Fermat's Spiral distribution is modeled for an unknown power magnitude, the overall efficiency and generated power also vary with the variation in the year's day (Fig. 12). Table 5 shows the power generated and the overall efficiency of the field.

**Fig. 11:** Attenuation plot of unoptimized Fermat's spiral distribution.

**Fig. 12:** Variation of Generated Power throughout the year for Fermat's Spiral Configuration Based on 4 Different Times of the Year (a) Vernal Eqvinox, (b) Autumnal Eqvinox, (c) Winter Solstice and (d) Summer Solstice.

**Table 5:** Generated Power of Heliostat Field based on Fermat's Spiral Distribution.

Day of the year	Power Generated (MW)	Mean (Overall Efficiency) (%)
Vernal Equinox	154.17	65.82
Summer Solstice	132.22	50.56
Autumnal Equinox	157.27	65.82
Winter Solstice	174.95	74.86

Notice that Fermat's spiral layout is performing better than radial staggered layout for a higher power magnitude. As explained in the succeeding articles, these layouts were further optimized for the given design location using the Genetic Algorithm.

It must be noted here that numerous conditions must be considered for calculating a particular field layout. However, it is the significance of existing literature in which it has been proved that by considering four days for the calculation of efficiency and performance of the field, a layout for the entire year can be generated. Hence, the final layout is generated based on only Vernal Equinox DNI values.

### 4.4 Optimization of the layouts

Both the layouts were optimized based on a predetermined range of values defined in the methodology chapter. Since the overall efficiency of the field varies throughout the year, the optimization was performed based on the average performance of both layouts on the days discussed in Table 3. Results of optimized field layouts based on radial staggered configuration are given in Fig. 13 (a). Table 6 shows the parameters and efficiency of the proposed field layout. A comparison of field performance before and after optimization is also presented in Table 6.

**Fig. 13:** Optimized Field Layout based on (a) Radial Staggered Arrangement and (b) Fermat's Spiral Distribution.

**Table 6:** Comparison between the performance of Fermat's Spiral and Radial Staggered Layouts.

Field Layout	Optimized Parameters				Generated Power (MW)	Mean efficiency before optimization (%)	Mean efficiency after optimization (%)	Required number of heliostats before optimization	Required number of heliostats after optimization
	TH (m)	WR	LH (m)	DS (m)					
Radial Staggered	61	1	12.6	0.16	50	74.72	83.24	957	523
Fermat's Spiral	72	1	12.5	0.14		65.82	80.44	864	541

After optimization, the number of heliostats required for generating the same power was reduced by 39.4 % (Table 4), and the overall efficiency was also increased by 8.52 %. It must be noted that the initial unoptimized layout was designed and analyzed based on an average value of four different days. However, the optimized layout is checked for average values of DNI on the same day of the year. This is done because, in heliostat field layout studies, the vernal equinox (which is used in our study) is taken as a reference point of the year. Fig. 13 (b) shows optimized Fermat's spiral distribution for the generation of field layout.

Although, Fermat's Spiral for a given day and DNI performed better than the Radial Stagger configuration for the given design point location of Quetta, Pakistan, and the same optimized parameters as used in radial stagger. However, after optimization, the number of heliostats required by the Radial Stagger arrangement outperformed the Fermat's Spiral. Table 6 shows the overall efficiency results of the optimization of this layout. It must be noted that in Fig. 13 (a), there are heliostats present along the symmetry axis that are not very large in number, but the algorithm suggested them to be placed in a manner that they can collide with each other. This issue is relevant to the security distance and blocking factor of the heliostats and is being investigated and an updated algorithm specifically addressing this scenario is still under development and will be published in near future as an extended version of this study. For Fig. 13 (b), the same issue persists and is being addressed separately.

## 5 Conclusion

The study presented the implementation of Genetic Algorithm for optimization of heliostat field layout for the local coordinates of Quetta, Balochistan. Radial Staggered and Fermat's Spiral heliostat field configurations for generation of 50 MW input thermal power were designed and compared. The following points were observed after analysis.

- Before optimization, Radial Staggered Field Layout generated 50 MW of thermal input power with an efficiency of 74.72 %.
- After the implementation of Genetic Algorithm, the thermal efficiency of Radial Staggered Field layout was improved by 8.52 % eventually attaining a value of 83.24 %.
- Before optimization, Fermat's Spiral Field Layout generated 50 MW of thermal input power with an efficiency of 65.82 % eventually attaining a value of 80.44 %.
- After the implementation of Genetic Algorithm, the thermal efficiency of Fermat's Spiral Field Layout was improved by 14.62 %.
- The increase in field efficiency also decreased the number of heliostats required to generate the same input power magnitude.
- Radial Staggered Field Layout required 523 heliostats to generate 50 MW input power after optimization while the number of heliostats decreased to 541 for Fermat's Spiral configuration.

This work provided a reference point to be initiated for the levelized cost of electricity analysis of central receiver-based systems in Quetta, Balochistan. As an extension of this study, a cost analysis encompassing the capital, infrastructure and operational cost optimization can be carried out which would unravel better horizons of renewable energy penetration in the national grid in general and energy deprived Balochistan in particular.

## Funding statement

The authors extend their appreciation to the Deputyship for Research & Innovation, Ministry of Education in Saudi Arabia for funding this research work through the project number 223202.

## Data availability statement

- Data associated with this study has not been deposited into a publicly available repository.
- Data will be made available on request.

## CRediT authorship contribution statement

**Muhammad Haris:** Writing – review & editing, Writing – original draft, Conceptualization. **Atiq Ur Rehman:** Writing – review & editing, Writing – original draft, Formal analysis. **Sheeraz Iqbal:** Writing – review & editing, Writing – original draft, Formal analysis. **Syed Owais Athar:** Writing – review & editing, Writing – original draft, Formal analysis, Data curation. **Hossam Kotb:** Writing – review & editing, Writing – original draft, Methodology, Formal analysis. **Kareem M. AboRas:** Writing – review & editing, Writing – original draft, Software, Formal analysis. **Abdulaziz Alkuhayli:** Data curation, Formal analysis. **Yazeed Yasin Ghadi:** Writing – review & editing, Writing – original draft, Data curation. **Kitmo:** Writing – review & editing, Writing – original draft, Supervision, Data curation.

## Declaration of competing interest

The authors declare that they have no known competing financial interests or personal relationships that could have appeared to influence the work reported in this paper.
